The article "Assessment of Expression of Regulatory T Cell Differentiation Genes in Autism Spectrum Disorder" was retracted in 2025. Reasons: compromised peer review; unreliable results or conclusions; citations of retracted work; concerns about the peer review.

# Assessment of Expression of Regulatory T Cell Differentiation Genes in Autism Spectrum Disorder

**DOI:** 10.3389/fnmol.2022.939224

**Published:** 2022-07-04

**Authors:** Mohammadarian Akbari, Reyhane Eghtedarian, Bashdar Mahmud Hussen, Solat Eslami, Mohammad Taheri, Seyedeh Morvarid Neishabouri, Soudeh Ghafouri-Fard

**Affiliations:** ^1^Skull Base Research Center, Loghman Hakim Hospital, Shahid Beheshti University of Medical Sciences, Tehran, Iran; ^2^Phytochemistry Research Center, Shahid Beheshti University of Medical Sciences, Tehran, Iran; ^3^Department of Pharmacognosy, College of Pharmacy, Hawler Medical University, Erbil, Iraq; ^4^Center of Research and Strategic Studies, Lebanese French University, Erbil, Iraq; ^5^Dietary Supplements and Probiotic Research Center, Alborz University of Medical Sciences, Karaj, Iran; ^6^Department of Medical Biotechnology, School of Medicine, Alborz University of Medical Sciences, Karaj, Iran; ^7^Institute of Human Genetics, Jena University Hospital, Jena, Germany; ^8^Department of Psychiatric, School of Medicine, Shahid Beheshti University of Medical Sciences, Tehran, Iran; ^9^Department of Medical Genetics, School of Medicine, Shahid Beheshti University of Medical Sciences, Tehran, Iran

**Keywords:** ASD, FLICR, MAFTRR, NEST, RMRP, TH2-LCR

## Abstract

Dysfunction of regulatory T cells (Tregs) has been shown to affect the etiology of autism spectrum disorder (ASD). Differentiation of this group of T cells has been found to be regulated by a group of long non-coding RNAs (lncRNAs). In this study, we have examined the expression of five lncRNAs that regulate this process in the blood samples of ASD cases compared with controls. These lncRNAs were FOXP3 regulating long intergenic non-coding RNA (FLICR), MAF transcriptional regulator RNA (MAFTRR), NEST (IFNG-AS1), RNA component of mitochondrial RNA processing endoribonuclease (RMRP), and Th2 cytokine locus control region (TH2-LCR). Expression of RMRP was significantly lower in total ASD cases compared to controls [expression ratio (95% CI) = 0.11 (0.08–0.18), adjusted *P*-value < 0.0001]. This pattern was also detected in both men and women cases compared with corresponding controls [expression ratio (95% CI) = 0.15 (0.08–0.29) and 0.08 (0.03–0.2), respectively]. Likewise, expression of NEST was reduced in total cases and cases among men and women compared with corresponding controls [expression ratio (95% CI) = 0.2 (0.14–0.28); 0.22 (0.12–0.37); and 0.19 (0.09–0.43), respectively; adjusted *P*-value < 0.0001]. Lastly, FLICR was downregulated in total cases and cases among both boys and girls compared with matched controls [expression ratio (95% CI) = 0.1 (0.06–0.19); 0.19 (0.08–0.46); and 0.06 (0.01–0.21), respectively; adjusted *P*-value < 0.0001]. These three lncRNAs had appropriate diagnostic power for differentiation of ASD cases from controls. Cumulatively, our study supports dysregulation of Treg-related lncRNAs in patients with ASD and suggests these lncRNAs as proper peripheral markers for ASD.

The article "Assessment of Expression of Regulatory T Cell Differentiation Genes in Autism Spectrum Disorder" was retracted in 2025. Reasons: compromised peer review; unreliable results or conclusions; citations of retracted work; concerns about the peer review.

## Introduction

Autism spectrum disorders (ASDs) delineate a diverse set of neurodevelopmental diseases described by deficits in social communicative skills accompanied by restrictive, monotonous, and stereotypic behaviors (American Psychiatric Association, 2013). This kind of disorder is estimated to affect approximately 1 in 54 people in the general population (Baxter et al., 2015). ASD has a complex background and an unidentified neurobiology which might be resulted from a multifaceted gene–environment interactive network (Barak and Feng, 2016; Ghafouri-Fard et al., 2019). Several lines of evidence indicate the importance of abnormal immune response in the etiopathogenesis of ASD (De Giacomo et al., 2021; Ellul et al., 2021). ASD has been associated with some immune-related disorders namely allergic conditions and psoriasis highlighting the presence of abnormal immune responses in these subjects (Zerbo et al., 2015). Others have reported inappropriate induction of immune cells, production of autoantibodies, and imbalances in cytokine levels in ASD cases (Gładysz et al., 2018).

Assessment of different types of immune cells in the blood of patients with ASD has shown a significant reduction in regulatory B cells and T cells in these patients vs. healthier controls, in spite of similar frequencies of B-cell memory and NK cells in these study groups (De Giacomo et al., 2021). Similarly, defects in CD4(+)CD25(high) regulatory T cells (Tregs) have been described in a significant number of ASD cases, leading to the autoimmune response in a subgroup of these patients (Mostafa et al., 2010). Moreover, a recent meta-analysis has indicated remarkable defects in CD4+ lymphocytes, particularly reduction of Tregs and surge in Th17 cells in patients with ASD supporting the importance of targeted immunotherapeutic approaches for this disorder (De Giacomo et al., 2021).

Non-coding RNAs have been revealed to be implicated in the regulation of Tregs differentiation and function (Luo and Wang, 2020; Ghafouri-Fard et al., 2022). Thus, dysregulation of these transcripts might participate in the etiology of disorders that are associated with impairment of Treg function. In the present study, we measured circulatory levels of five long non-coding RNAs (lncRNAs) which have been found to affect the differentiation of T cells in patients with ASD. These lncRNAs are FOXP3 regulating long intergenic non-coding RNA (FLICR), MAF transcriptional regulator RNA (MAFTRR), NEST (IFNG-AS1), RNA component of mitochondrial RNA processing endoribonuclease (RMRP), and Th2 cytokine locus control region (TH2-LCR).

The article "Assessment of Expression of Regulatory T Cell Differentiation Genes in Autism Spectrum Disorder" was retracted in 2025. Reasons: compromised peer review; unreliable results or conclusions; citations of retracted work; concerns about the peer review.

## Materials and Methods

### Patients and Controls

A total of 30 ASD cases (11 girls and 19 boys) and 41 healthy children (11 girls and 30 boys) were enlisted. Blood samples were gathered from all patients with ASD and control children. Cases were assessed in the university-affiliated centers from 2018 to 2019, based on the Diagnostic and Statistical Manual of Mental Disorders (American Psychiatric Association, 2013). Moreover, we used the Autism Diagnostic Observation Schedule-Generic (ADOS-G) for further assessment of ASD cases (Lord et al., 2000). None of the cases and controls had structural brain diseases or systemic disorders. Written informed consent was obtained from guardians of all children. The study protocol was permitted by the Ethics Committees of Shahid Beheshti University of Medical Sciences.

### Expression Assays

Total RNA was retrieved from specimens by using the commercial RNA Isolation Kit (PicoPure™, Thermo Fisher Scientific) based on the details described in the kit manual. Then, RNA was converted to cDNA by using the Smobio kit (Taiwan). The expression of Treg-associated lncRNAs was quantified in all samples using the qRT-PCR kit (GeneDireX, Miaoli County, Taiwan). All experiments were performed in duplicate. Each PCR run included a negative control (no template control). LightCycler^®^ 96 (Roche Life Science) instrument was used for expression assays. Table 1 demonstrates the information about primers. *B2M* was used as the normalizer.

**TABLE 1:** Primer sequences.

Gene	Sequence 5 → 3	Primer length (bp)
*B2M*	F-AGATGAGTATGCCTGCCGTG	20
	R-GCGGCATCTTCAAACCTCCA	20
*FLICR*	F-GGG CTT TTC CAG AAG GGT CT	20
	R-AGC CCA GGG TTC TAG TCG	18
*MAFTRR*	F-CTG AAG GGA CAG GAC GGA CAA C	22
	R-GGG GAA AAC CTG GAA AGA GGG A	22
*NEST*	F-AGC TGA TGG CAA TCT	21
	R-TGA CTT CTC CAG CGT TTT	21
*RMRP*	F-GTA GAC ATT CCC CGC TTC CCA	21
	R-GAG AAT GAG CCC CGT GTG GTT	21
*TH2-LCR*	F-GCT CCC CAG GCT TTT GAG ATA	21
	R-TGG TGA TGC TGA AGG GAG AC	20

### Statistical Analysis

Statistics were assessed using GraphPad Prism version 9 (GraphPad Software, La Jolla, CA, United States). Expression levels of five Treg-related genes were measured in the blood of patients with ASD and healthy controls. The expression of each gene was calculated using the following formula:


Efficiency⁢adjusted⁢Ct⁢of⁢B2M-Efficiency⁢adjusted⁢Ct⁢of⁢target⁢gene

Shapiro–Wilk test was used for evaluation of normal/Gaussian distribution of values. An unpaired *t*-test or non-parametric test (Mann–Whitney *U* test) was used to recognize differentially expressed lncRNAs between subgroups. The effect of disease and gender on the expression of lncRNAs was assessed using two-way ANOVA and Tukey *post hoc* tests in each subgroup.

The article "Assessment of Expression of Regulatory T Cell Differentiation Genes in Autism Spectrum Disorder" was retracted in 2025. Reasons: compromised peer review; unreliable results or conclusions; citations of retracted work; concerns about the peer review.

Box and whisker plots were designed to show −delta Ct values. Median (line), mean (cross), interquartile range (box), and minimum and maximum values were demonstrated in these figures.

Correlations between gene expression levels in both study groups were measured using Spearman’s rank correlation coefficient since some values were not normally distributed.

The receiver operating characteristic (ROC) curves were used to evaluate the diagnostic power of transcript levels of differentially expressed genes. The optimum threshold was obtained using Youden’s J parameter. *P*-value < 0.05 was considered significant.

## Results

General information about ASD cases and controls is shown in Table 2.

**TABLE 2:** General demographic data of enrolled cases and controls.

Study groups	Parameters	Values	
Patients	Sex (number)	Male	19
		Female	11
	Age (years, mean ± SD)	Male	6 ± 1.33
		Female	6 ± 1.73
Controls	Sex (number)	Male	30
		Female	11
	Age (years, mean ± SD)	Male	6.2 ± 1.88
		Female	5.63 ± 1.28

### Expression Assays

Expression levels of RMRP, NEST, and FLICR were significantly different between ASD cases and controls (Figure 1). However, there was no significant difference in the expression of TH2-LCR and MAFTRR transcripts between subgroups.

**FIGURE 1:** Relative expressions of five Treg-related genes RMRP, TH2LCR, NEST, and FLICR genes in patients with ASD (total) and healthy controls (total) as designated by –delta Ct values. –Delta Ct data were plotted as box and whisker plots. Median, mean, and interquartile ranges are shown. Unpaired *t*-test or non-parametric test (Mann–Whitney *U* test) was used to identify differentially expressed genes between two groups (****P-value < 0.0001; ns, non-significant).

Then, we assessed the expression of these genes in different sex-based subgroups of patients (Figure 2). We detected a significant effect of disease factors on expression levels of RMRP, NEST, and FLICR lncRNAs in subgroups. Besides, we detected a significant effect of sex factor on expression levels of RMRP and NEST in subgroups. Finally, the interaction of sex and disease factors had significant effects on the expression level of the FLICR gene in subgroups.

**FIGURE 2:** Relative expression levels of five Treg-related genes in subgroups of patients with ASD vs. control subgroups as described by –delta Ct values. –Delta Ct data is plotted. Median, mean, and interquartile ranges are shown. The effects of disease and gender on the expression of lncRNAs were appraised using two-way ANOVA and Tukey *post hoc* tests (^****^P-value < 0.0001; ns, non-significant).

The article "Assessment of Expression of Regulatory T Cell Differentiation Genes in Autism Spectrum Disorder" was retracted in 2025. Reasons: compromised peer review; unreliable results or conclusions; citations of retracted work; concerns about the peer review.

Expression of RMRP was significantly lower in entire ASD cases compared with control children [expression ratio (95% CI) = 0.11 (0.08–0.18), adjusted *P*-value < 0.0001]. This pattern was also detected in both male and female cases compared with corresponding controls [expression ratio (95% CI) = 0.15 (0.08–0.29) and 0.08 (0.03–0.2), respectively]. Likewise, expression of NEST was lower in total cases and in cases among male and female, compared with corresponding control subjects [expression ratio (95% CI) = 0.2 (0.14–0.28); 0.22 (0.12–0.37) and 0.19 (0.09–0.43), respectively; adjusted *P*-value < 0.0001]. Lastly, FLICR was downregulated in total cases and cases among boys and girls compared with corresponding controls [expression ratio (95% CI) = 0.1 (0.06–0.19); 0.19 (0.08–0.46) and 0.06 (0.01–0.21), respectively; adjusted *P*-value < 0.0001]. Table 3 demonstrates the detailed statistics of expression study of five Treg related genes in patients with ASD compared with healthy controls.

**TABLE 3:** The results of the expression study of five Treg-related genes in peripheral blood of patients with ASD compared with healthy controls (^&^, adjusted *P*-value, RE, expression ratio).

Studied genes		Total patients vs. total controls (30 vs. 41)	Male patients vs. normal males (19 vs. 30)	Female patients vs. normal females (11 vs. 11)
RMRP	ER (95% CI)	0.11 (0.08–0.18)	0.15 (0.08–0.29)	0.08 (0.03–0.2)
	P^&^	<0.0001*	<0.0001*	<0.0001*
TH2LCR	ER (95% CI)	1.23 (0.7–2.24)	1.2 (0.47–3.34)	1.29 (0.31–5.27)
	P^&^	0.47	0.91	0.96
NEST	ER (95% CI)	0.2 (0.14–0.28)	0.22 (0.12–0.37)	0.19 (0.09–0.43)
	P^&^	<0.0001*	<0.0001*	<0.0001*
FLICR	ER (95% CI)	0.1 (0.06–0.19)	0.19 (0.08–0.46)	0.06 (0.01–0.21)
	P^&^	<0.0001*	<0.0001*	<0.0001*
MAFTRR	ER (95% CI)	0.78 (0.35–1.8)	0.68 (0.18–2.54)	1.67 (0.24–11.3)
	P^&^	0.49	0.87	0.89

*P-value at a significance level of P < 0.05.

Significant correlations have been detected between several pairs of Treg-related lncRNAs in both study groups (Table 4).

**TABLE 4:** Spearman’s correlations between transcript levels among the patients with ASD (*N* = 30) and healthy controls (*N* = 41).

	TH2LCR		NEST		FLICR		MAFTRR	
	Patients	Control	Patients	Control	Patients	Control	Patients	Control
RMRP	0.31	0.7**	0.46*	0.62**	0.54*	−0.2	0.17	0.61**
TH2LCR			0.08	0.53**	0.65**	−0.18	0.71**	0.66**
NEST					0.39*	−0.3	0.2	0.45*
FLICR							0.61**	−0.06

*P-value at a significance level of P < 0.05.

**P-value at a significance level of P < 0.001.

The article "Assessment of Expression of Regulatory T Cell Differentiation Genes in Autism Spectrum Disorder" was retracted in 2025. Reasons: compromised peer review; unreliable results or conclusions; citations of retracted work; concerns about the peer review.

We also evaluated the diagnostic power of differentially expressed genes between ASD cases and controls (Figure 3).

**FIGURE 3:** Receiver operating characteristic curves of RMRP, IFNG-AS1, and FLICR lncRNAs transcript levels show their diagnostic power in the differentiation of total ASD cases from controls.

Ribonucleic component of mitochondrial RNA processing endoribonuclease had the best AUC values in the separation of total ASD cases from total controls (AUC ± SD = 0.97 ± 0.01) and in the separation of female and male cases from corresponding controls (AUC ± SD = 1 ± 0 and 0.97 ± 0.02, respectively). Moreover, the AUC values of NEST were 0.96 ± 0.02, 0.9 ± 0.07, and 0.97 ± 0.01 in total cases, among male and female cases compared with corresponding controls, respectively. Finally, these values were 0.89.04, 0.93 ± 0.05, and 0.86 ± 0.06 for FLICR, respectively (Table 5).

**TABLE 5:** The results of ROC curve analysis in total patients with ASD as well as sex-based subgroups.

	RMRP				NEST				FLICR			
	AUC ± SD	Sensitivity	Specificity	*P*-value	AUC ± SD	Sensitivity	Specificity	*P*-value	AUC ± SD	Sensitivity	Specificity	*P*-value
Total patients vs. total normal controls (30 vs. 41)	0.97 ± 0.01	0.97	0.88	<0.0001	0.96 ± 0.02	0.96	0.85	<0.0001	0.89 ± 0.04	0.77	0.93	<0.0001
Female patients vs. female normal controls (11 vs. 11)	1 ± 0.00	1	1	<0.0001	0.9 ± 0.07	0.9	0.9	0.001	0.93 ± 0.05	0.81	1	0.0006
Male patients vs. male normal controls (18 vs. 30)	0.97 ± 0.02	0.95	0.93	<0.0001	0.97 ± 0.01	0.95	0.9	<0.0001	0.86 ± 0.06	0.74	0.93	<0.0001

## Discussion

Regulatory T cells have a crucial role in self-tolerance since they decrease autoimmune reactions through the suppression of proinflammatory responses (Dasgupta et al., 2020). Dysfunction or reduction of these cells has been detected in a number of autoimmune disorders, namely multiple sclerosis (Zozulya and Wiendl, 2008) and rheumatoid arthritis (Toubi et al., 2005). The function and differentiation of Tregs are modulated by lncRNAs. For instance, FLICR has been found to control the expression of Foxp3, leading to the generation of a group of Tregs with decreased expression of FoxP3. Notably, a certain polymorphism within the *FoxP3* gene has been previously shown to affect the risk of ASD in the Iranian population (Safari et al., 2017). This lncRNA has a particular effect in IL-2 deficiency conditions. Mechanistically, FILCR alters chromatin structure in a particular district of the Foxp3 locus to limit the activity of Tregs. This lncRNA enhances the development of autoimmune diabetes but confines antiviral response (Zemmour et al., 2017). TH2-LCR is another transcript with an important role in the modulation of immune responses. This lncRNA controls the expression of TH2 cytokines, modulates chromatin structure at the TH2 cytokine locus, and is involved in the pathoetiology of allergic asthma (Koh et al., 2010). Another lncRNA contributing to the modulation of immune response is NEST. This lncRNA binds to WDR5, a constituent of the H3K4 methyltransferase complex which can modify H3 methylation at the *IFN-G* locus, thus affecting IFN-γ levels (Gomez et al., 2013). This lncRNA reduces the expression of CD40L and TFT-bet in CD4+ T cells, thus reducing TH1-enhanced proliferation of Treg cells (Luo et al., 2017). MAFTRR is a chromatin-associated lncRNA with particular expression in TH1 cells. Decreased expression of this lncRNA leads to differentiation of T cells toward the TH2 phenotype (Ranzani et al., 2015). Finally, lncRNA RMRP has been shown to influence TH17 cell effector functions in association with DDX5 (Huang et al., 2015). It is worth mentioning that although TH17 and Treg cells have different functional properties, they have similar developmental requirements. Actually, a number of regulators, namely TGF-β, IL-6, and ATRA regulate the differentiation of antigen-naïve T-cells to either TH17 or Tregs (Omenetti and Pizarro, 2015).

The article "Assessment of Expression of Regulatory T Cell Differentiation Genes in Autism Spectrum Disorder" was retracted in 2025. Reasons: compromised peer review; unreliable results or conclusions; citations of retracted work; concerns about the peer review.

In brief, we have reported downregulation of RMRP, NEST, and FLICR lncRNAs in the peripheral circulation of ASD cases compared with controls. This observation highlights abnormal regulation of T cell functions in the circulation of these patients and suggests this mechanism as a possible underlying cause in the neurobiology of ASD. However, the exact mechanism of participation of these lncRNAs in the pathoetiology of ASD needs to be elucidated.

Most notably, these three lncRNAs, particularly RMRP were found to be sensitive and specific markers for ASD. This finding broadens our current knowledge in biomarker discovery for ASD and potentiates these lncRNAs as therapeutic targets for this disorder. Subsequent expression assays in postmortem brain tissues or cerebrospinal fluid samples would be useful for confirmation of our results. Moreover, our study lacks functional assays.

## Data Availability Statement

The raw data supporting the conclusions of this article will be made available by the authors, without undue reservation.

## Ethics Statement

The study protocol was permitted by the Ethics Committees of Shahid Beheshti University of Medical Sciences. Written informed consent to participate in this study was provided by the participants’ legal guardian/next of kin.

## Author Contributions

SG-F wrote the draft and revised it. MT designed and supervised the study. SE analyzed the data. SN, RE, BH, and MA collected the data and performed the experiment. All authors read and contributed to the article and approved the submitted version.

The article "Assessment of Expression of Regulatory T Cell Differentiation Genes in Autism Spectrum Disorder" was retracted in 2025. Reasons: compromised peer review; unreliable results or conclusions; citations of retracted work; concerns about the peer review.

## Conflict of Interest

The authors declare that the research was conducted in the absence of any commercial or financial relationships that could be construed as a potential conflict of interest. The reviewer SA-J declared a past co-authorship with the authors to the handling editor.

## Publisher’s Note

All claims expressed in this article are solely those of the authors and do not necessarily represent those of their affiliated organizations, or those of the publisher, the editors and the reviewers. Any product that may be evaluated in this article, or claim that may be made by its manufacturer, is not guaranteed or endorsed by the publisher.
